# iMPT-FDNPL: Identification of Membrane Protein Types with Functional Domains and a Natural Language Processing Approach

**DOI:** 10.1155/2021/7681497

**Published:** 2021-10-11

**Authors:** Wei Chen, Lei Chen, Qi Dai

**Affiliations:** ^1^College of Information Engineering, Shanghai Maritime University, Shanghai 201306, China; ^2^College of Life Sciences, Zhejiang Sci-Tech University, Hangzhou 310018, China

## Abstract

Membrane protein is an important kind of proteins. It plays essential roles in several cellular processes. Based on the intramolecular arrangements and positions in a cell, membrane proteins can be divided into several types. It is reported that the types of a membrane protein are highly related to its functions. Determination of membrane protein types is a hot topic in recent years. A plenty of computational methods have been proposed so far. Some of them used functional domain information to encode proteins. However, this procedure was still crude. In this study, we designed a novel feature extraction scheme to obtain informative features of proteins from their functional domain information. Such scheme termed domains as words and proteins, represented by its domains, as sentences. The natural language processing approach, word2vector, was applied to access the features of domains, which were further refined to protein features. Based on these features, RAndom k-labELsets with random forest as the base classifier was employed to build the multilabel classifier, namely, iMPT-FDNPL. The tenfold cross-validation results indicated the good performance of such classifier. Furthermore, such classifier was superior to other classifiers based on features derived from functional domains via one-hot scheme or derived from other properties of proteins, suggesting the effectiveness of protein features generated by the proposed scheme.

## 1. Introduction

Membrane protein refers to the protein that can bind to the cell membrane and is an important part of the cell membrane. It exposes a surface that is very suitable for merging to the membrane [1]. There are lots of membrane proteins in human. They perform various functions related to cell survival. About 30% of genes can encode membrane proteins [2], 60% of membrane proteins can be used as drug targets, and some membrane proteins can act as enzyme mediators in the immune system [3]. It is reported that the function of membrane protein is highly associated with its type. Identification of the types of membrane proteins is an important step to uncover their functions. Traditional experimental methods can provide solid results. However, they have some evident defects, such as low efficiency and high cost. The large-scale tests for identification of membrane protein types via these methods are almost impossible. Thus, it is urgent to design quick and cheap methods.

In recent years, lots of new computational methods have proposed, providing strong technical support for designing classifiers for identification of membrane protein types. On the other hand, several online databases have been set up for collecting various information of proteins, giving strong data support. To date, several classifiers have been proposed to identify membrane protein types. Most classifiers are based on machine learning algorithms. These classifiers always learn patterns based on the information of membrane proteins, whose types have been determined. These patterns can be used to determine the types of given proteins. Several existing classifiers used features extracted from protein sequences [4–9]. Amino acid composition (AAC) and pseudo amino acid composition (PseAAC) are two classic schemes to access features from protein sequences. Functional domains are also used to build classifiers for identification of membrane protein types [10–12]. The classifiers incorporating such information always provided good performance. However, the usage of functional domain information is still at a low level. One-hot scheme was used to encode proteins based their functional domain information. Through this scheme, each protein was encoded into a binary vector, where each component represented one domain. If the domain was annotated on a given protein, its corresponding component was set to one; otherwise, it was set to zero. However, such scheme had some evident defects. For example, the performance of the classifiers was quite sensitive to some domains. This study gave an investigation on the usage of functional domain information of proteins.

In this study, we set up a novel classifier to identify membrane protein types. This classifier adopted the novel features obtained from functional domain information of proteins via a natural language processing approach, word2vector. These features were fed into a multilabel classification scheme, RAndom k-labELsets (RAKEL) [13], to set up the classifier. Classic classification algorithm, random forest (RF) [14], was selected as the base classifier in RAKEL. The proposed classifier was called iMPT-FDNPL. The tenfold cross-validation indicated the good performance of such classifier. It was also superior to other classifiers that were constructed with other widely used feature extraction schemes, including the classifier using features derived from functional domain information via one-hot scheme.

## 2. Materials and Methods

### 2.1. Database

The data of human membrane proteins was sourced from Huang et al.'s study (dataset S1) [15]. 2883 membrane proteins, encoded by UniProt IDs, were obtained. In fact, these proteins were extracted from a larger dataset retrieved from the UniProt database (release 2012_09) [16] by using CD-HIT [17]. The sequence similarity of any two proteins was smaller than 0.7. These 2883 proteins were classified into six types: (1) GPI- (glycosyl phosphatidyl isohydrin-) anchored, (2) lipid-anchor, (3) multipass, (4) peripheral, (5) single-channel type I, and (6) single-pass II type [18]. Because we adopted functional domain information to encode proteins, those without such information were excluded. 2729 membrane proteins remained. These proteins were still classified into six abovementioned types. The distribution of 2729 membrane proteins on six types is shown in Table 1. The sum of protein numbers in all six types was 2810 (last row of Table 1), which was bigger than the number of different proteins. It was suggested that some proteins belonged to more than one types. As shown in Figure 1, 73 proteins belonged to two types, 4 proteins belonged to three types, whereas rest proteins belonged to one type. Thus, it is a multilabel classification problem to assign types to membrane proteins.

### 2.2. Feature Engineering

Feature engineering is an important step in designing efficient classifiers. In this study, we should extract features from each membrane protein, which can retain essential properties of proteins. Functional domain is widely used to investigate various protein-related problems, including membrane protein type prediction. The classic way to employ such information is one-hot scheme. Several classifiers have been built with such scheme, and they provided good performance [10–12]. As mentioned above, such scheme also had some defects. Here, we proposed a new scheme to adopt functional domain information, thereby encoding membrane proteins in a new way.

#### 2.2.1. Domain Representation

The functional domain information of all human proteins was retrieved from the InterPro database (http://ftp.ebi.ac.uk/pub/databases/interpro/, accessed in February 2021) [19]. 17,410 IPR terms were annotated on 171,472 human proteins. In this study, we adopted a natural language processing approach to analyze this information. To this end, IPR terms were deemed as words and proteins, represented by one or more IPR terms, were termed as sentences. Accordingly, the well-known word2vector method was applied on them to learn a feature vector for each IPR term. This study used the word2vector program obtained from https://github.com/RaRe-Technologies/gensim. Default parameters were adopted.

#### 2.2.2. Protein Representation

As mentioned above, the feature vector of each IPR term was learnt by word2vector. Based on them, we can further access the feature vectors of proteins. Here, a simple way was adopted. The feature vector of a given protein was defined as the average vector of feature vectors of IPR terms that was annotated on such protein. For example, for a certain protein A4D1S5, there are three IPR terms, say IPR001806, IPR005225, IPR027417, and the average vector of three vectors, representing above three IPR terms, respectively, was used to represent A4D1S5.

### 2.3. Multilabel Classifier

This study adopted a problem transformation method, RAKEL [13], to build the multilabel classifier, which has wide applications in dealing with several biological and medicine problems [20–27]. From the original multilabel classification problem, several single-label classification problems are derived as follows. Given a problem with *l* labels, denoted by *L*_1_, *L*_2_, ⋯, *L*_*l*_, it first randomly constructs *m* label subsets, each of which contains *k* labels, where 1 ≤ *k* ≤ *l*. For each label subset, members in its power set are deemed as new labels. Samples are assigned new labels according to their original labels. For example, for the label subset {*L*_1_, *L*_2_, *L*_3_}, the labels of each sample are first restricted to this subset, i.e., labels in this subset are picked up and the rest are discarded. Then, the remaining labels are put together as a new label. If the labels for one sample are *L*_1_, *L*_2_ and *L*_4_, *L*_1_  and *L*_2_ are first selected and {*L*_1_, *L*_2_}, a member of the power set of {*L*_1_, *L*_2_, *L*_3_}, is assigned to such sample as its new label. Accordingly, each sample has exactly one new label. Then, a classifier can be built with a given base single-label classifier. The *m* label subsets induce *m* single-label classifiers. The final multilabel classifier integrates these single-label classifiers. In detail, given a query sample, each single-label classifier provides its prediction. Such prediction can be refined to the binary predictions for labels involved in this classifier. For each label, the binary predictions yielded by classifiers involving this label are selected and count the proportion of classifiers that predict this label. If this proportion is higher than a predefined threshold, which is always set to 0.5, the label is assigned to the query sample.

To quickly implement the RAKEL algorithm, we used the tool “RAKEL” in Meka [28], retrieved from http://waikato.github.io/meka/. Several values of *m* and *k*, the main parameters of RAKEL, were tried in this study. For convenience, the classifiers built by RAKEL were termed as RAKEL classifiers.

### 2.4. Base Classifier

The multilabel classifier built by RAKEL needs a base single-label classifier as mentioned above. One of the most classic algorithms, RF [14], was selected in this study. It is an ensemble classifier, consisting of several decision trees. Each decision tree is constructed by randomly selecting samples and features. Given a sample, each decision tree provides its prediction. RF counts these predictions and determines the final prediction using majority voting. Although decision tree is quite weak, RF is much more robust. Thus, it is always an important candidate to build classifiers for tackling different problems [29–39].

In this study, we adopted the tool “RandomForest” integrated in Meka [28], which implements RF.

### 2.5. Performance Measurement

All classifiers were assessed by tenfold cross-validation [40–44]. This method randomly and equally divides samples into ten subsets. Each subset is singled out to constitute the test set one by one, and rest subsets are put together to constitute the training set. Accordingly, each sample is predicted only once.

After obtaining the outcomes of tenfold cross-validation, we calculated three measurements to assess the quality of results, including exact matching, accuracy, and hamming loss [25–27], which can be computed by

(1) $$\begin{array}{c} \left\{\begin{array}{c} \text{Exact match}=\frac{1}{n}\overset{n}{\underset{i=1}{\sum }}\nabla \left(L_{i},L_{i}^{\prime }\right),\\ \text{Accuracy}=\frac{1}{n}\overset{n}{\underset{i=1}{\sum }}\left(\frac{\left\|L_{i}\cap L_{i}^{\prime }\right\|}{\left\|L_{i}\cup L_{i}^{\prime }\right\|}\right),\\ \text{Hamming loss}=\frac{1}{n}\overset{n}{\underset{i=1}{\sum }}\left(\frac{\left\|L_{i}∆L_{i}^{\prime }\right\|}{m}\right), \end{array}\right. \end{array}$$

where *n* denotes the overall number of samples, *m* stands for the number of labels (*m* = 6 in this study), *L*_*i*_ and *L*_*i*_′ represent the set of true labels and predicted labels of the *i*^th^ sample, respectively,Δ stands for the set symmetric difference operation, and ∇ is defined as follows:

(2) $$\begin{array}{c} \nabla \left(L_{i},L_{i}^{\prime }\right)=\left\{\begin{array}{cc} 1 & \text{If }{\text{L}}_{i}\text{ is identifical to }{\text{L}}_{i}^{\prime },\\ 0 & \text{Otherwise}. \end{array}\right. \end{array}$$

Obviously, the higher exact matching and the accuracy, the better the performance of the classifier. For hamming loss, the lower the hamming loss, the better the performance. For easy comparisons, an integrated measurement, called integrated score, was defined as below

(3) $$\begin{array}{c} \text{Integrated score}=\text{exact match}*\text{accuracy}*\left(1-\text{hamming loss}\right). \end{array}$$

The higher the score, the better the classifier.

## 3. Results and Discussion

In this study, we set up a multilabel classifier, iMPT-FDNPL, for prediction of membrane protein types. Such classifier employed the features derived from functional domain information of proteins. The entire procedures are shown in Figure 2. In this section, we would give the evaluation results and comparisons with other classifiers.

### 3.1. Performance of iMPT-FDNPL

iMPT-FDNPL adopted the features derived from functional domain information via word2vector. Because the optimum dimension of features was unknown, several dimensions were tried, including dimensions from 50 to 500 with interval 50. Furthermore, the main parameter *m* in RAKEL was set to 10, and another main parameter *k* was set to all integers between 2 and 6. As for the parameter of RF, number of decision trees, it was set to integers from 100 to 500 with interval 100. RAKEL classifiers with all possible parameter settings were set up and assessed by tenfold cross-validation. The outcomes showed that when the dimension was set to 350, *k* = 6, *m* = 10, and the number of decision trees was 500, the RAKEL classifiers provided the highest integrated score of 0.6874. Thus, this classifier was the proposed multilabel classifier, iMPT-FDNPL. The exact match, accuracy, and hamming loss were 0.851, 0.853, and 0.053, respectively, which are listed in Table 2. The exact match and accuracy both exceed 0.850, suggesting the good performance of iMPT-FDNPL.

To fully assess the performance of iMPT-FDNPL under tenfold cross-validation, 20 additional tenfold cross-validations on this classifier were conducted. The obtained values of exact matching, accuracy, hamming loss, and integrated score are illustrated in Figure 3. We can see that exact match varied from 0.853 to 0.860, accuracy from 0.856 to 0.863, hamming loss from 0.049 to 0.052, and integrated score from 0.6921 to 0.7058. Above four measurements varied in a small interval, implying that the performance of iMPT-FDNPL was quite stable no matter how samples were divided.

### 3.2. Comparison of RAKEL Classifiers with Other Base Classifiers

The proposed classifier, iMPT-FDNPL, adopted RF as the base classifier. In fact, we also attempted another classic classification algorithm, support vector machine (SVM) [45]. Similar to RF, the tool “SMO” integrated in Meka was directly employed in this study, which implements one type of SVM, whose training procedures are optimized by the sequential minimal optimization algorithm [46, 47]. The kernel was polynomial kernel or RBF kernel. Various values of regularization parameter *C* were tried, including 1, 2, 3, and 4. The exponent of polynomial kernel was set to 1, 2, 3, and 4. As for parameter *γ* of RBF kernel, it was set to various values between 0.01 and 0.05. The feature dimensions and *m*, *k* in RAKEL were the same as those in Section 3.1. All RAKEL classifiers with possible parameter settings were built and evaluated by tenfold cross-validation. The best performance (highest integrated score) of RAKEL classifiers with SVM using two different kernels is listed in Table 2. If the basic classifier was SVM (polynomial kernel), the integrated score was 0.6515, exact match was 0.831, accuracy was 0.834, and hamming loss was 0.060. If SVM (RBF kernel) was the base classifier, the integrated score was 0.6787, exact match was 0.846, accuracy was 0.848, and hamming loss was 0.054. The comparisons of those yielded by iMPT-FDNPL indicated that the proposed classifier was superior to these RAKEL classifiers. It was proper to select RF as the base classifier to construct the classifier.

### 3.3. Comparison of BR Classifiers

In this study, we adopted RAKEL to build the multilabel classifier. Here, another multilabel classifier construction method, Binary Relevance (BR) [48], was employed to build the classifiers. Similar to RAKEL, it also needs one base classifier. We still used three base classifiers mentioned above: RF, SVM with polynomial kernel, and SVM with RBF kernel. We tried the same parameter settings as those in above sections. With all possible parameter settings, several classifiers were set up and assessed by tenfold cross-validation. For convenience, these classifiers were called BR classifiers.

The best performance of BR classifiers with different base classifiers is listed in Table 2. The integrated scores of these BR classifiers were 0.5778, 0.6152, and 0.6544, respectively, which were all lower than that of the iMPT-FDNPL. Furthermore, the exact match and accuracy of iMPT-FDNPL were also higher than the corresponding measurements of three BR classifiers. As for hamming loss, iMPT-FDNPL provided lower performance than BR classifier with SVM (RBF kernel) as the base classifier. However, the hamming loss of iMPT-FDNPL was lower than those of other two BR classifiers. All these results indicated the superiority of the iMPT-FDNPL. In addition, given a base classifier, RAKEL classifiers always provided higher performance than BR classifiers, implying RAKEL was more powerful to construct multilabel classifiers for identifying membrane protein types than BR.

### 3.4. Comparison of Classifiers with Other Embedding Features

In this study, the multilabel classifier, iMPT-FDNPL, adopted features derived from functional domains via a natural language processing approach to encode membrane proteins. As mentioned above, one-hot scheme is a more widely used way to encode proteins. Here, each protein was encoded by such scheme. Then, the RAKEL and BR were employed to construct classifiers, and the base classifier was SVM or RF. With all possible parameter settings used above, several classifiers were built, each of which was assessed by tenfold cross-validation. The best performance for RAKEL and BR with one of the base classifiers is listed in Table 3, from which we can see that with such features, the RAKEL with SVM (polynomial kernel) provided the best performance. In detail, the integrated score was 0.6794, and three measurements (exact match, accuracy, and hamming loss) were 0.847, 0.848, and 0.054. Such performance was lower than that of the iMPT-FDNPL. Thus, features derived from functional domains via word2vector were more efficient than the features derived from functional domains via one-hot scheme for identifying membrane protein types.

Gene ontology (GO) [49] and KEGG pathway [50] information was also widely used to investigate protein- or gene-related problems. With the similar procedures that were done for functional domains, GO terms and pathways were termed as words, whereas proteins, annotated by GO terms and pathways, were considered as sentences. We can obtain feature vectors of GO terms and pathways via word2vector. Then, a membrane protein was represented by an average vector of vectors of GO terms and pathways that were annotated on such protein. Likewise, several dimensions from 50 to 500 with interval 50 were generated. RAKEL or BR with SVM or RF as the base classifier was employed. Several classifiers were constructed with all possible parameter settings. All classifiers were evaluated by tenfold cross-validation. Similarly, the best performance using RAKEL or BR with one base classifier is listed in Table 4. Evidently, in this case, RAKEL with SVM (polynomial kernel) generated the highest performance with integrated score of 0.6106. The exact match was 0.808, accuracy was 0.810, and hamming loss was 0.067. The exact match, accuracy, and integrated score were all lower than those of iMPT-FDNPL, and the hamming loss was larger than that of iMPT-FDNPL. These results indicated that features derived from functional domains via word2vector were more powerful to identify membrane protein types than those derived from GO and pathways via the same natural language processing approach. It was also implied that functional domain information was more related to membrane protein types than GO and pathway information.

Network embedding algorithm is a type of recently proposed computational methods, which can abstract associations of nodes in one or more networks and extract a feature vector for each node. It has also been applied to process some protein-related problems [25, 26, 34, 51–55]. Here, we used such method to extract protein features. To this end, eight protein networks were first built according to protein-protein interaction information reported in STRING (https://www.string-db.org/, version 10.0) [56]. The network embedding algorithm, Mashup [53], was applied on these networks to access the feature vectors of proteins. The dimensions included integers from 50 to 500 with interval 50. Obtained feature vectors of membrane proteins were fed into RAKEL or BR with SVM or RF as the base classifier to build the classifiers. All possible parameter settings used above were tried, and all constructed classifiers were assessed by tenfold cross-validation.  Table 5 lists the best performance of RAKEL or BR classifiers with different base classifiers. Interestingly, the RAKEL with SVM (polynomial kernel) also provided the best performance. The integrated score of such classifier was 0.6054. Other three measurements were 0.805, 0.807, and 0.068, respectively. However, compared with the performance of iMPT-FDNPL (see Table 2), such performance was still lower. These results also suggested the effectiveness of features derived from functional domain via word2vector for prediction of membrane protein types.

With above arguments, we can conclude that features derived from functional domain via word2vector are quite effective to identify membrane protein types because classifiers based such features were more powerful than those based on other three types of features, which were derived from functional domain via one-hot scheme, from GO and pathway via word2vector, and from protein network via Mashup, respectively. To further confirm the superiority of features derived from functional domain via word2vector, the best classifiers using above three types of features were further evaluated by tenfold cross-validation for 20 times. Obtained values of exact match, accuracy, hamming loss, and integrated score are shown in Figure 4. For easy comparisons, those of the classifier (iMPT-FDNPL) using features derived from functional domain via word2vector are also shown in this figure. It is easy to observe that iMPT-FDNPL always generated highest exact match, accuracy, and integrated score and lowest hamming loss. All these further confirmed the superiority of the used features, which was the main reason why iMPT-FDNPL can provide such good performance.

## 4. Conclusions

This study sets up a multilabel classifier, iMPT-FDNPL, to identify membrane protein types. A novel feature extraction scheme was integrated in this classifier, which can extract efficient protein features by applying a natural language processing approach, word2vector, to functional domain information of proteins. The cross-validation results showed that such classifier was quite powerful and superior to classifiers using other types of protein features. Such results also indicated the superiority of features extracted by the proposed scheme. It is hopeful that such classifier can be a useful tool to identify membrane protein types, and the novel feature extraction scheme can be used to tackle other protein-related problems. All codes and data are available athttps://github.com/mufei111/iMPT-FDNPL.

## Figures and Tables

**Figure 1:** An illustration to show the distribution on the number of types a membrane belongs to. Four membrane proteins belong to three types, 73 proteins belong to two types, and rest 2652 proteins belong to one type.

**Figure 2:** Entire procedures to construct and evaluate the multilabel classifier, iMPT-FDNPL. Membrane proteins and types are retrieved from the UniProt database. The types are termed as labels. Function domain information is obtained from the InterPro database. This information is processed by a natural language processing approach (word2vector), and the outcomes are used to encode proteins. Labels and vectors are fed into RAKEL with random forest as the base classifier to construct the multilabel classifier. This classifier is evaluated by tenfold cross-validation.

**Figure 3:** Boxplot to show the performance of iMPT-FDNPL using tenfold cross-validation for 20 times. (a) Accuracy; (b) exact match; (c) hamming loss; (d) integrated score. Each measurement varies in a same range.

**Figure 4:** Boxplot to show the performance of classifiers with different feature types using tenfold cross-validation for 20 times. (a) Accuracy; (b) exact match; (c) hamming loss; (d) integrated score. Features derived from functional domain via word2vector are most efficient to identify membrane protein types.

**Table 1:** Distribution of membrane proteins on six types.

Membrane protein type	Number of proteins
GPI-anchor	69
Lipid-anchor	211
Multipass	1306
Peripheral	530
Single-pass type I	539
Single-pass type II	155
Total	2810

**Table 2:** Performance of different multilabel classifiers with features derived from functional domain information via a natural language processing approach.

Scheme (base classifier)	Exact match	Accuracy	Hamming loss	Integrated score
RAKEL (RF) (iMPT-FDNPL)	0.851	0.853	0.053	0.6874
RAKEL (SVM-polynomial kernel)	0.831	0.834	0.060	0.6515
RAKEL (SVM-RBF kernel)	0.846	0.848	0.054	0.6787
BR (RF)	0.781	0.782	0.054	0.5778
BR (SVM-polynomial kernel)	0.804	0.815	0.061	0.6152
BR (SVM-RBF kernel)	0.829	0.831	0.050	0.6544

**Table 3:** Performance of different multilabel classifiers with features derived from functional domain information via one-hot scheme.

Scheme (base classifier)	Exact match	Accuracy	Hamming loss	Integrated score
RAKEL (RF)	0.825	0.827	0.061	0.6406
RAKEL (SVM-polynomial kernel)	0.847	0.848	0.054	0.6794
RAKEL (SVM-RBF kernel)	0.846	0.847	0.054	0.6778
BR (RF)	0.785	0.788	0.049	0.5882
BR (SVM-polynomial kernel)	0.774	0.778	0.049	0.5726
BR (SVM-RBF kernel)	0.836	0.840	0.048	0.6685

**Table 4:** Performance of different multilabel classifiers with features derived from gene ontology and pathway information via a natural language processing approach.

Scheme (base classifier)	Exact match	Accuracy	Hamming loss	Integrated score
RAKEL (RF)	0.761	0.762	0.083	0.5324
RAKEL (SVM-polynomial kernel)	0.808	0.810	0.067	0.6106
RAKEL (SVM-RBF kernel)	0.808	0.810	0.068	0.6099
BR (RF)	0.584	0.584	0.087	0.3113
BR (SVM-polynomial kernel)	0.717	0.738	0.068	0.4931
BR (SVM-RBF kernel)	0.747	0.755	0.063	0.5284

**Table 5:** Performance of different multilabel classifiers with features derived from protein networks via a network embedding algorithm.

Scheme (base classifier)	Exact match	Accuracy	Hamming loss	Integrated score
RAKEL (RF)	0.758	0.759	0.085	0.5264
RAKEL (SVM-polynomial kernel)	0.805	0.807	0.068	0.6054
RAKEL (SVM-RBF kernel)	0.801	0.803	0.070	0.5981
BR (RF)	0.584	0.584	0.088	0.3110
BR (SVM-polynomial kernel)	0.712	0.730	0.068	0.4844
BR (SVM-RBF kernel)	0.746	0.756	0.063	0.5284

## Data Availability

The original data used to support the findings of this study are available at the UniProt database.
